The article "Protective Effect of D-Limonene against Oxidative Stress-Induced Cell Damage in Human Lens Epithelial Cells via the p38 Pathway" was retracted in 2022. Reasons: errors in the images; duplicated images; overlap with earlier publications.

# Protective Effect of D-Limonene against Oxidative Stress-Induced Cell Damage in Human Lens Epithelial Cells via the p38 Pathway

**DOI:** 10.1155/2016/5962832

**Published:** 2015-11-23

**Authors:** Jie Bai, Yi Zheng, Gang Wang, Ping Liu

**Affiliations:** ^1^Key Laboratory of Harbin Medical University Eye Center, Eye Hospital, First Affiliated Hospital, Harbin Medical University, Harbin 150001, China; ^2^State Key Laboratory of Veterinary Biotechnology, Harbin Veterinary Research Institute, Chinese Academy of Agricultural Sciences, Harbin 150001, China

## Abstract

Oxidative stress, as mediated by ROS, is a significant factor in initiating the development of age-associated cataracts; D-limonene is a common natural terpene with powerful antioxidative properties which occurs naturally in a wide variety of living organisms. It has been shown to have antioxidant effect; we found that D-limonene can effectively prevent the oxidative damage caused by H_2_O_2_ and propose that the main mechanism underlying the inhibitory effects of D-limonene is the inhibition of HLECs apoptosis. In the present study, we used confocal-fluorescence microscopy, flow cytometry analysis, Hoechst staining, H_2_DCFDA staining, transmission electron microscopy, and immunoblot analysis; the results revealed that slightly higher concentrations of D-limonene (125–1800 *μ*M) reduced the H_2_O_2_-induced ROS generation and inhibited the H_2_O_2_-induced caspase-3 and caspase-9 activation and decreased the Bcl-2/Bax ratio. Furthermore, it inhibited H_2_O_2_-induced p38 MAPK phosphorylation. Thus, we conclude that D-limonene could effectively protect HLECs from H_2_O_2_-induced oxidative stress and that its antioxidative effect is significant, thereby increasing the cell survival rate.

## 1. Introduction

Oxidative stress, as mediated by ROS, is a major factor in the aging process. It is widely recognized that the intraocular generation of oxygen free radicals is a significant factor initiating the development of age-associated cataracts [1–5]. Exposure to oxidative stress can lead to lens opacification in both experimental animal models and cultured lens systems [6–8]. Oxidative stress is also known to activate mitogen-activated protein kinases (MAPKs), including stress-activated p38 mitogen-activated protein kinase (p38 MAPK), extracellular signal-regulated kinase (ERK), and c-Jun N-terminal kinase (JNK). The MAPK pathway plays important roles in proliferation and apoptosis of HLECs induced by various stimuli [6, 9–11]. The findings of recent studies suggest that early cataract treatments should focus on rescuing HLECs from oxidative damage.

The epithelial layer of the lens is the main target of the oxidative insult and any external insult may affect its antioxidant status. Apoptosis of HLECs is suggested to be a cause of cataract formation. Apoptosis is a well-known mechanism of cell death that plays critical roles in a variety of biological systems, including the initiation and progression of cataracts [11–14]. The relationship between oxidative stress and apoptosis has been widely studied, and an increase in ROS generation has long been associated with the apoptotic response [15].

Age-related cataracts are currently among the leading causes of severe visual impairment. This visual impairment, and the consequent disability and reduction in quality of life, significantly impacts patients' mental health. Cataract extraction is one of the most frequent day-case procedures to correct vision loss. However, it presents a large financial burden on the national health care system, mandating the search for pharmaceutical agents that can prevent or delay the onset of cataracts.

D-limonene is a common natural terpene with powerful antioxidative properties that occurs naturally in a wide variety of living organisms. It has been shown to have antioxidant, antitumorigenic, and anti-inflammatory properties, and it plays an important role in gallstone drainage* in vitro* and* in vivo* [16–21]. Many studies have demonstrated that D-limonene can eliminate oxygen free radicals and protect organisms from oxidative damage [19, 20, 22]. It has even been shown to protect normal lymphocytes from oxidative stress related diseases, including cancer [20]. However, its protective effect against oxidative stress in relation to inhibition on HLECs apoptosis has not yet been reported.

Based on previous studies, we anticipated that the antioxidant properties of D-limonene could protect the human lens from the oxidative stress that induces cataract development and this terpene could be beneficial for treating cataracts.

## 2. Materials and Methods

### 2.1. Reagents and Antibodies

D-limonene with 97% purity was purchased from Sigma Company (USA). Stock solutions were diluted to the desired final concentration with medium just prior to use. Hoechst 33342 was purchased from Invitrogen (USA). Dulbecco's modified Eagle's medium (DMEM) was purchased from Gibco (Grand Island, NY). Annexin V and propidium iodide (PI) were obtained from Becton Dickinson (Mountain View, CA). 2′,7′-Dichlorofluorescein diacetate (H_2_DCFDA) and a bicinchoninic acid (BCA) protein assay kit were obtained from Beyotime (Beyotime Institute of Biotechnology, China). Anti-Bax, anti-Bcl-2, anti-caspase-3, anti-caspase-9, anti-p38 MAPK, and anti-phosphorylated p38 MAPK (P-p38) antibodies were purchased from Santa Cruz Biotechnology Inc. (Santa Cruz, CA, USA).

### 2.2. Cell Cultures

HLECs (ATCC, America) were maintained in a humidified atmosphere of 5% CO_2_ in DMEM supplemented with 20% fetal bovine serum (FBS), penicillin (100 U/mL), and streptomycin (100 *μ*g/mL) at 37°C. The cells were routinely subcultured every 2-3 days.

### 2.3. Assessment of Cell Viability

Cells were cultured at a density of 2 × 10^4^ cells per well in 96-well microplates with 2% FBS overnight, then the medium was removed, and fresh DMEM without serum was added to the plates. After 30 minutes of incubation, they were pretreated with various concentrations of D-limonene (62.5, 125, 250, 500, 1000, and 2000 *μ*M) for 12, 24, and 48 h and were then treated with H_2_O_2_ for 24 hours. Finally, the cell survival was measured using an MTT assay. Briefly, for the MTT assay, 100 *μ*L MTT solution (0.5 mg/mL in phosphate-buffered saline; PBS) was added to each well. After incubating for 1 h, the MTT solution was removed and DMSO was added to dissolve the dye. The absorbency was measured at 450 nm using a microplate reader and a background control as the blank. The cell survival ratio was expressed as a percentage of the control. The control cells were only starved and were not exposed to H_2_O_2_.

### 2.4. Morphologic Changes of Apoptotic Cells Detected by Confocal-Fluorescence Microscopy

The HLECs, as before, were grown in 2% FBS overnight at 37°C. The medium was removed and fresh DMEM without serum was added to the plates. After 30 min of incubation, the cells were treated with different concentrations of H_2_O_2_ for 24 h. The cells were then fixed in 4% paraformaldehyde in PBS (pH 7.4) for 30 min. After fixation, they were washed twice with PBS and were then stained with Hoechst 33342 (Hoechst/Propidium Iodide Cell Staining Kit, BIPEC BIOREAGENT) for 15 min at room temperature. After being washed in PBS and then resuspended, 1 mL of each of buffer A and then PI was added, and the solution was incubated for 15 min. The cells were immediately examined with a fluorescence microscope (Olympus Optical Co. Ltd., Japan). An excitation wavelength of 488 nm was used for observation.

### 2.5. Detection of Cell Apoptosis by Flow Cytometry

Cells were plated and incubated in a six-well plate at 1 × 10^5^ cells per well and were then treated with D-limonene at different concentrations (0 (as control), 62.6, 125, 250, 500, 1000, or 2000 *μ*M) for 12 h. Next, the cells were incubated in the presence or absence of H_2_O_2_ (a single dose of 100 *μ*M H_2_O_2_) at 37°C for 24 h. After the 24 h, they were then washed twice with phosphate-buffered saline (PBS) and harvested by digestion with trypsin in the absence of EDTA. The cells were collected and microfuged at 2000 rpm for 5 min. The culture fluids were discarded, 5 *μ*L of annexin V-FITC and 10 *μ*L of PI were added to the cell pellet at room temperature and the samples were incubated in the dark for 15 min. The samples were then gently shaken and analyzed using Cell-Quest software (Becton Dickinson, Mountain View, CA) with the FL1-H and FL2-H channels.

### 2.6. Hoechst 33342

The percentage and morphology of the apoptotic cell nuclei were analyzed using a Hoechst 33342 staining protocol. Briefly, the cells were stained with 10 *μ*g/mL Hoechst 33342 under dark conditions at room temperature for 30 min. After washing three times with PBS, the nuclear morphology of the stained cells was examined under a fluorescence microscope with an excitation of 485 nm and an emission of 530 nm. The nonspecific fluorescence values in the absence of cells were subtracted from the fluorescence values.

### 2.7. Reactive Oxygen Species Detection

The intracellular accumulation of ROS was investigated using the fluorescent dye H_2_DCFDA, which is converted to dichlorofluorescein diacetate (DCF), a membrane impermeable and highly fluorescent compound in the presence of ROS. The cells were incubated in 10 *μ*M H_2_DCFDA for 20 min at 37°C and then washed twice with PBS. The fluorescence intensity of DCF was detected using a fluorescence microscope (Leica DMI 4000, German).

### 2.8. Morphologic Changes of Apoptotic Cells Detected by Electronic Microscopy

Cells were treated and fixed with 2.5% phosphate-buffered glutaraldehyde overnight and then postfixed in 1% cold phosphate-buffered osmium tetroxide for 1 h. After rinsing with PBS, the cells were embedded in fresh resin, sectioned, double stained with uranyl acetate and lead citrate, and examined under a transmission electron microscope (H-7650 JEM-1200EX, Japan).

### 2.9. Real-Time PCR

Total RNA was extracted from cells using an RNA Kit (Omega, United States) according to the manufacturer's instructions. cDNA was synthesized according to the RNA PCR kit protocol (Takara, Dalian, China). Real-time PCR was performed in a reaction with a total volume of 20 *μ*L using SYBR Premix Ex Taq II (TaKaRa, Dalian, China). The reaction conditions were 95°C for 5 min, followed by 40 cycles of 95°C for 5 s, 55°C for 30 s, and 72°C for 30 s. *β*-actin was used as an internal control for sample normalization. The data are expressed relative to the control level. The primers used in this study are listed in Table 1.

### 2.10. Western Blot Analysis

Cells were washed twice with ice-cold PBS and lysed in 100 *μ*L of RIPA buffer (1 mM PMSF, 1% NP-40, 50 mM Tris-HCl (pH 7.2), 2 mM EDTA, and 100 mM NaCl). Cell lysates were centrifuged at 4°C for 10 min at 12,000 ×g, the supernatant was collected, and the protein concentration was evaluated using a BCA protein assay kit (Beyotime Institute of Biotechnology, China). 20 *μ*g of protein extract was separated on 12% SDS–PAGE gels and transferred onto nitrocellulose membranes (Millipore, USA) at 20 V for 23 minutes. The membranes were blocked in 5% nonfat dry milk for 1 h at room temperature, and washes were performed using TBS buffer. The membranes were incubated in primary antibody overnight at 4°C and then incubated in the corresponding peroxidase-linked secondary antibody at room temperature for 1 h. Protein bands were detected using a standard enhanced chemiluminescence method following the manufacturer's protocol (Amersham).

### 2.11. Statistical Analysis

All statistical analyses were performed using SPSS (version 10.0). The data were expressed as the mean ± standard error means (SEM) for the indicated number of separate experiments. The statistical analysis of the data was performed using Student's *t*-test. *P* < 0.05 was considered statistically significant. All of the experiments were performed at least three times.

## 3. Results

### 3.1. The Preventive Effect of D-Limonene against Oxidative Stress-Induced Damage of HLECs

As shown in Figure 1(a), H_2_O_2_ impaired the cell viability in a dose- and time-dependent manner. The morphology of the HLECs changed following treatments with different concentrations of H_2_O_2_ (Figures 1(b) and 1(c)). Confocal-fluorescence microscopy showed nuclear apoptosis when HLECs were exposed to H_2_O_2_ at concentrations of higher than 100 *μ*M (Figure 1(c)). Viability of cells treated with D-limonene was not significantly affected at any of the tested concentrations (Figure 1(d)). Therefore, under our test conditions, it was safe to treat HLECs with up to 2000 *μ*M D-limonene for 48 h. Pretreating cells with D-limonene prevented H_2_O_2_-induced oxidative stress damage to HLECs in a dose- and time-dependent manner, as shown in Figure 1(e).

### 3.2. D-Limonene Protects HLECs against H_2_O_2_-Induced Apoptosis

The annexin V/PI double staining method was used to evaluate the protective effect of D-limonene against H_2_O_2_-induced cell apoptosis. As shown in Figure 2(a), there was an increase in the number of PI single-positive cells (indicative of mainly necrotic cells) after treating HLECs with 100 *μ*M H_2_O_2_. The number of annexin V single-positive cells (indicative of mainly apoptotic cells) was decreased following D-limonene treatment in a dose-dependent manner (Figure 2(b)). To confirm the flow cytometry data on H_2_O_2_-induced apoptotic cell death, we examined the number of Hoechst-positive HLECs following D-limonene treatment. As expected, the number of these cells increased after 100 *μ*M H_2_O_2_ treatment (Figure 3(a)), which resulted in 40.00 ± 4.26% apoptotic cells in HLECs compared with 3.50 ± 0.29% apoptotic control cells (Figure 3(b)). The percentage of Hoechst-positive cells was closely correlated with the number of annexin V-positive cells in Figure 2(a).

### 3.3. D-Limonene Inhibit H_2_O_2_-Induced ROS Generation in HLECs

There was a lack of staining in the H_2_O_2_-free control group, as expected (Figure 4). HLECs that were only exposed to H_2_O_2_ were heavily stained, indicating that there was a marked increase in ROS levels. This increase in intracellular ROS, however, was prevented by pretreating cells with D-limonene in a concentration-dependent manner. This finding indicates that D-limonene can prevent the generation of intracellular ROS in HLECs challenged with H_2_O_2_.

### 3.4. Changes in Cell Morphology and Membrane Integrity Detected by Transmission Electron Microscope (TEM)

Figure 5 shows ultrastructural changes in HLECs exposed to H_2_O_2_. The ultrastructures of control cells and 1000 *μ*M D-limonene-treated cells were normal, with intact nuclei and healthy-looking mitochondria and Golgi bodies. In contrast, H_2_O_2_-treated HLECs displayed an irregular nuclear outline, condensed chromosomes in apoptotic cells, a loose endoplasmic reticulum, and morphologically abnormal mitochondrial structures. In the presence of increased concentrations of H_2_O_2_, the cell membranes were not intact, the cytoplasm was swollen, the nucleus was pyknotic, and apoptotic bodies appeared. In addition, the cytoplasm showed significant vacuolization. These findings were well correlated with the observed effect on confocal-fluorescence microscopy (Figure 1(c)). In D-limonene-pretreated HLECs, the cellular ultrastructure appeared to be improved compared with that of cells treated with 100 *μ*M H_2_O_2_ alone. Essentially, the transmission electron microscopic observations indicated that D-limonene could preserve the cellular ultrastructural changes induced by H_2_O_2_.

### 3.5. D-Limonene Inhibits the Expression of Caspase-3 and Caspase-9 and Modulates the Expression of Bcl-2 Family Proteins, as Induced by H_2_O_2_ in HLECs

To investigate the possible mechanism by which D-limonene inhibits HLECs apoptosis, western blot and real-time PCR analyses were performed. As shown in Figure 6, the protein and mRNA expression levels of antiapoptotic Bcl-2 were downregulated in the H_2_O_2_-treated group compared with the control untreated group (*P* < 0.05), whereas the protein and mRNA expression levels of proapoptotic Bax, caspase-3, and caspase-9 were upregulated in the H_2_O_2_-treated group compared with the control untreated group (*P* < 0.05). The D-limonene treatment, however, prevented the H_2_O_2_-induced upregulation of Bax and downregulation of Bcl-2. These results were confirmed by determining the Bcl-2/Bax ratio (Figure 6(c)). These findings also suggest that D-limonene inhibits HLECs apoptosis through a mechanism that utilizes the pathways involving Bcl-2, Bax, caspase-3, and caspase-9.

### 3.6. Effect of D-Limonene on the Phosphorylation of p38 in HLECs in Response to H_2_O_2_

As shown in Figure 7(a), D-limonene inhibited the phosphorylation of p38, in the presence and absence of H_2_O_2_. Although no change in the total p38 protein level was observed, H_2_O_2_-induced p38 phosphorylation (lane 1) was significantly inhibited in D-limonene-treated cells (lane 2) (*P* < 0.01). Furthermore, pretreatment for 30 min with SB203580 (10 *μ*M), a specific inhibitor of p38 kinase, abolished the p38 phosphorylation induced by H_2_O_2_. These results indicated that the pretreatment with D-limonene and SB203580 inhibited H_2_O_2_-induced p38 MAPK activity.

## 4. Discussion and Conclusion

Cataracts significantly impair daily function and quality of life in activities such as reading, walking, and driving. Cataract patients with low visual acuity or blindness may experience adverse consequences, both at an individual and at a public level. Reduced visual sensitivity impairs judgment of environmental hazards and thereby increases anxiety related to mobility and accidents. Patients with cataracts are associated with depression and anxiety symptoms that lead to social and psychological problems. The symptoms generate a loss of self-esteem and of occupational status, resulting in a loss of income.

Oxidative stress is widely recognized to play an important role in the pathogenesis of cataract development. Oxidative stress induced by H_2_O_2_ is believed to be a key cause of cell dysfunction [3]. Previous studies have demonstrated that H_2_O_2_-induced HLECs apoptosis is a traditional model for studying cataractogenesis [23–25]. H_2_O_2_ contains active oxygen, can permeate cellular membrane, and can enter the cell and cause additional membrane damage. Increased concentrations of H_2_O_2_ have also been found in aqueous humor from cataract patients [2].

In our study, we found that H_2_O_2_ can cause apoptosis (Figures 1(b), 1(c), 2, 3, and 5) and can significantly increase ROS levels (Figure 4) in HLECs. Cell viability also decreased as the concentration of and incubation time in H_2_O_2_ increased (Figure 1(a)). The cell viability significantly increased, however, when cells were pretreated with D-limonene (Figure 1(e)). Treating cells with D-limonene at concentration ranging from 62.5 to 2000 *μ*M attenuated the H_2_O_2_-induced loss of cell viability without any significant negative effects on viability and it was found to be relatively safe for HLECs up to a concentration of 2000 *μ*M (Figure 1(d)). These findings indicate that D-limonene can effectively prevent the oxidative damage caused by H_2_O_2_, thereby increasing the cell survival rate. Flow cytometry analysis (Figure 2) and Hoechst assay (Figure 3) also showed that the H_2_O_2_-induced HLECs apoptosis was significantly reduced when cells were pretreated with D-limonene. Based on these results, we propose that the main mechanism underlying the inhibitory effects of D-limonene is the inhibition of HLECs apoptosis.

Limonene is an essential component in citrus oil. D-limonene (1-methyl-4-(1-methylethenyl) cyclohexene), the most common isomer of limonene, is considered to have a relatively low toxicity. Once orally administered, it is rapidly and almost completely absorbed by the gastrointestinal tract in both humans and animals [26]. Studies have shown that D-limonene does not pose carcinogenic or mutagenic nephrotoxic risks to humans [27]. Several* in vitro* and* in vivo* studies have shown that D-limonene has antioxidative, antitumorigenic, anti-inflammatory, and antinociceptive properties [19–21]. Although the protective effects of D-limonene have been reported in various models, very little is known about its antioxidant activity in relation to apoptosis-related cataracts. Therefore, we aimed to determine whether D-limonene plays a protective role against H_2_O_2_-induced injury in HLECs.

The relationship between oxidative stress and apoptosis has been widely studied, and an increase in ROS generation has long been associated with cell apoptosis [16–18, 22]. To determine whether suppressing ROS production prevents apoptosis, we examined the caspase family. Some studies have shown that HLECs treated with H_2_O_2_ exhibit high expression levels of caspase-3 and caspase-9 [9, 25, 28]. Consistent with these results, we also found in our study that H_2_O_2_-induced apoptosis is accompanied by an increase in the expression levels of caspase-9 and caspase-3 at the protein and RNA levels. However, these elevated expression levels were reduced in the D-limonene-treated group compared with the H_2_O_2_-treated group (Figure 6).

Bcl-2 family members play an important role in regulating apoptosis. These proteins are either antiapoptotic (e.g., Bcl-2, Bcl-XL, and Mcl-1) or proapoptotic (e.g., Bax, Bak, and Bad) [29], and the interactions among them may influence cell fate. Bax and Bcl-2 are considered to be the principal factors that determine whether the process of apoptosis proceeds by activating caspases. The ratio of Bcl-2 to Bax proteins is critical for determining whether apoptosis occurs. A decrease in this ratio promotes the release of cytochrome c from the mitochondria into the cytosol, leading to the subsequent activation of caspase-9 and caspase-3 [30]. In this study, we found that the Bcl-2/Bax ratio was significantly lower in cells treated with H_2_O_2_ and that this decrease was prevented by pretreating cells with D-limonene (Figure 6). These results indicate that Bcl-2 family proteins may play critical role in regulating the H_2_O_2_-induced apoptosis in HLECs and that D-limonene protects against H_2_O_2_-induced apoptosis by regulating the expression levels of Bcl-2 and Bax.

Oxidative stress can modulate phosphorylated MAPK levels, which have been shown to play a role in cataractogenesis [31, 32]. Several studies have reported that D-limonene reduces oxidative stress in various types of cells by inhibiting the MAPK signaling cascade [20]. Multiple members of the kinase families in this pathway can be activated by protein phosphorylation and p38 MAPK plays key roles in cellular apoptosis and death [31]. To detect the pathways that are involved in the protective role of D-limonene against oxidative stress, we examined the expression of this major signaling protein in the MAPK pathway.

Our findings show that H_2_O_2_-induced apoptosis is mainly mediated through the activation of p38 MAPK and that D-limonene inhibits the phosphorylation of p38 MAPK (Figure 7). These findings are consistent with those of our previous studies [6, 10]. We found that D-limonene inhibits the H_2_O_2_-stimulated activation of the p38 MAPK signaling pathway, and thus, it may be an effective natural drug for the treatment of cataracts due to its effects on ameliorating oxidative damage to HLECs.

The relationship between oxidative stress and cataracts has been widely studied. However, until now, there have been no effective clinical methods for preventing HLECs' apoptosis induced by oxidative stress. An important intracellular signaling pathway that leads to ROS-mediated apoptosis helps activate caspases. D-limonene, a potent antioxidant, can effectively prevent oxidative damage by regulating the expression of caspase-3, caspase-9, Bax, and Bcl-2 and by inhibiting the phosphorylation of p38 MAPK. The short-term effect of D-limonene is mainly antiapoptotic. The cell-protective effect of D-limonene so as to attenuate apoptotic cell death requires further study to elucidate a mechanism. Therefore, we hypothesized that such protective effects might directly involve the antioxidant properties of D-Limonene. Further research is necessary to establish the role of D-limonene as a potential antioxidant related to its effect on the activity of a cell's antioxidant enzymes, such as catalase, peroxidase, and superoxide dismutase.

In conclusion, D-limonene effectively protects HLECs from H_2_O_2_-induced oxidative stress, increases cell viability by reducing ROS generation, and suppresses apoptosis by inhibiting the activation of caspases in HLECs. D-limonene can also regulate the expression of Bax and Bcl-2 and inhibit the phosphorylation of p38 MAPK. These findings suggest that this terpene may be an important compound that can be used in the development of new agents for the effective treatment of cataracts.

## Figures and Tables

**Figure 1:** D-limonene reduced H_2_O_2_-induced cell death in HLECs. (a) HLECs were incubated in 25–800 *μ*M of H_2_O_2_ for 12, 24, and 48 h. (b) Morphology of HLECs exposed to H_2_O_2_ (0–800 *μ*M) for 24 h. (c) HLECs are shown to be stained with the nuclear dye Hoechst 33342 (blue)/PI (red) and photographed by a confocal-fluorescence microscope. (d) HLECs were incubated in 62.5–2000 *μ*M of D-limonene for 12, 24, and 48 h. (e) HLECs were pretreated with various concentrations of D-limonene (62.5–2000 *μ*M) for 12 h, 24 h, and 48 h and then incubated in the presence of 100 *μ*M H_2_O_2_ for 24 h. The results were measured by an MTT assay and expressed as a percentage of the untreated control.

**Figure 2:** D-limonene inhibited H_2_O_2_-induced apoptosis in HLECs. (a) Annexin V/PI staining of HLECs incubated in 500, 1000, and 2000 *μ*M D-limonene for 12 h and then treated with 100 *μ*M H_2_O_2_ for 24 h is shown. The percentage of cells in each of the four quadrants is shown inside of each area. (b) The quantitative analysis of the apoptosis rate in HLECs is shown. ^*∗*^ *P* < 0.05, ^*∗∗*^ *P* < 0.01.

**Figure 3:** Protective effect of D-limonene against H_2_O_2_–induced apoptosis. HLECs were pretreated with 1000 *μ*M D-limonene for 12 h and then treated with 100 *μ*M H_2_O_2_ for 24 h. The cells were then stained with Hoechst 33342 and observed using a fluorescence microscope. (a) Morphological apoptosis was observed using an inverted microscope. Cells that were exposed to H_2_O_2_ exhibited morphological changes typical of apoptosis, such as chromatin condensation and nuclear shrinkage. (b) The statistical analysis of the nuclear morphological change is shown. At least 70 cells in three different fields were counted per well in three separate experiments. ^*∗∗*^ *P* < 0.01.

**Figure 4:** Effect of D-limonene on H_2_O_2_-induced generation of ROS in HLECs. Cells were treated with 100 *μ*M H_2_O_2_ for 2 h after incubation in the absence or presence of D-limonene for 24 h. After this treatment, the production of ROS was determined using 10 *μ*M H_2_DCFDA. The morphological features were observed using fluorescence microscopy.

**Figure 5:** HLECs were photographed by an electronic microscope. Cells that were exposed to H_2_O_2_ (100, 400, and 800 *μ*M) for 24 h exhibited morphologic changes typical of apoptosis, such as cell shrinkage, irregular nuclear outline, chromatin condensation, apoptotic body, and cytoplasm vacuolization. In the D-limonene-pretreated HLECs, the cellular ultrastructure appeared to be more improved than that of cells treated with 100 *μ*M H_2_O_2_ alone.

**Figure 6:** D-limonene inhibits H_2_O_2_-induced caspase-3 and caspase-9 activation and modulates the expression of Bcl-2 family proteins in HLECs. The cells were pretreated with 500 and 1000 *μ*M D-limonene for 12 h and then exposed to 100 *μ*M H_2_O_2_ for 24 h. (a) The protein expression levels of Bax, Bcl-2, caspase-3, and caspase-9 were analyzed by western blot analysis; quantitative analysis was performed by measuring intensity relative to the untreated control. (b) The real-time PCR analysis of the apoptosis factors is shown. (c) The Bcl-2/Bax ratio was assessed. Each value represents the mean ± SEM for three independent experiments. ^*∗*^ *P* < 0.05, ^*∗∗*^ *P* < 0.01.

**Figure 7:** Effect of D-limonene on the expression of P-p38 in HLECs in response to H_2_O_2_. The cells were incubated with 1000 *μ*M D-limonene for 24 h with/without pretreatment with 10 *μ*M SB203580 for 30 min before 100 *μ*M H_2_O_2_ incubation for 1 h. (a) Phosphorylation of protein was measured by western blot using phospho-p38 MAPK antibody (lane 1). Total p38 MAPK protein was also measured using anti-p38 MAPK antibody (lane 2). Representative blots for three independent experiments are shown. (b) Quantitative analysis was performed by measuring intensity relative to the untreated control. ^*∗∗*^ *P* < 0.01.

**Table 1:** Primer sequences used in real-time PCR experiments.

Name		Sequence (5′-3′)
Bax	Forward	AAGCTGAGCGAGTGTCTCAAGC
363 bp	Reverse	CGCCACAAAGATGGTCACG
Bcl-2	Forward	GTACATCCATTATAAGCTGTCGCAG
363 bp	Reverse	AAGAGCTCCTCCACCACCGT
Caspase-3	Forward	AGCACTGGAATGACATCTCGGT
350 bp	Reverse	GTCTCAATGCCACAGTCCAGTTC
Caspase-9	Forward	CTACGAGAACGATGACGAGTGCT
237 bp	Reverse	CTCTCGAGGAAGGCCACGTA
*β*-actin	Forward	GGGTCAGAAGGATTCCTATG
237 bp	Reverse	GGTCTCAAACATGATCTGGG

## Abbreviations

ROS: Reactive oxygen species
HLECs: HLECs
H_2_O_2_: Hydrogen peroxide
p38 MAPK: p38 mitogen-activated protein kinase
ERK: Extracellular signal-regulated kinase
JNK: c-Jun N-terminal kinase
H_2_DCFDA: 2′, 7′-Dichlorofluorescein diacetate
BCA: Bicinchoninic acid
DMEM: Dulbecco's modified Eagle's medium
FBS: Fetal bovine serum.
